# An Immune-Related Genetic Feature Depicted the Heterogeneous Nature of Lung Adenocarcinoma and Squamous Cell Carcinoma and Their Distinctive Predicted Drug Responses

This article has been retracted.

**DOI:** 10.1155/2022/8447083

**Published:** 2022-08-27

**Authors:** Qiuyuan Li, Yan Jiang, Nan Song, Bin Zhou, Zhao Li, Lei Lin

**Affiliations:** Department of Thoracic Surgery, Tongji University Shanghai Pulmonary Hospital, No. 507 Zhengmin Rd., Shanghai, China

## Abstract

One of the primary causes of global cancer-associated mortality is lung cancer (LC). Current improvements in the management of LC rely mainly on the advancement of patient stratification, both molecularly and clinically, to achieve the maximal therapeutic benefit, while most LC screening protocols remain underdeveloped. In this research, we first employed two algorithms (ESTIMATE and xCell) to calculate the immune/stromal infiltration scores. This helped identify the altered immune infiltration landscapes in lung adenocarcinoma (LUAD) and squamous cell carcinoma (LUSC). Afterward, based on their immune-related characteristics, we successfully stratified the LUAD and LUSC into 2 and 3 clusters, respectively. Different from the conventional bioinformatic approaches that start from the investigation of differential expression of single genes, differentially enriched curated gene sets identified through gene set variation analyses (GSVA) were curated, and gene names were reconstructed afterward. Furthermore, weighted gene correlation network analyses (WGCNA) were used to reveal hub genes highly connected with the clustering process. Actual expression levels of critical hub genes among different clusters were compared and so were the functional pathways these genes enriched into. Lastly, a computational method was applied to predict and compare the responses of each cluster to primary therapeutic agents. The heterogeneity presented in our study, along with the drug responses expected for identified clusters, may shed light on future exploration of combination immunochemotherapy that facilitates the optimization of individualized therapy.

## 1. Introduction

Globally, lung cancer (LC) is a highly prevalent malignancy. In 2020, there were an estimated 2,206,771 new LC cases in both sexes, occupying 11.4% of all new cancer diagnoses worldwide that year. As the second most prevalent cancer, second only to breast cancer, LC has the highest cancer mortality and the worst age-standardized mortality rate (ASR) of 18 per 100,000 (GLOBOCAN 2020, https://gco.iarc.fr/today). In the USA, the 5-year survival rate for LC is as low as 6% in patients with metastasis, and metastasis is present in 57% of patients [1]. Gene set variance analysis (GSVA) is a method for the unsupervised classification of samples [2]. In contrast to traditional schemes, GSVA features a gene set of interest, allowing the relative enrichment of a specific gene set in a sample population to be quantified [2, 3]. GSVA can reveal subtle changes in pathway activity in different groups with greater stability and sensitivity.

Non-small-cell lung cancer (NSCLC) comprises the predominant type of LC, which could be further classified into adenocarcinoma (LUAD), squamous cell carcinoma (LUSC), and large cell neuroendocrine carcinoma. In contrast to LUSC, which arises from airway basal epithelial cells, adenocarcinoma generally originates locally from Clara cells, type II pneumocytes, or mucin-producing cells, and it compromises the majority of NSCLC [27413711, 34354223]. However, such crude stratification is far from enough to satisfy the need to provide an individualized treatment strategy. Thus, in addition to a set of currently available screening or diagnostic tools, there is an urgent need to update patient stratification at a molecular level for better therapeutic advantages. Various attempts have been done to try to hierarchically cluster patients/tumors into subsets with distinctive molecular or genetic characteristics as available expression and somatic mutation profiles expand [4–6]. Clinically, agents targeting relatively actionable alterations have been applied towards defined groups of patients, especially those at an advanced stage, which include inhibitors of EGFR [7, 8], ALK [9–11], ROS1 [12, 13], and PD-1/PD-L1 [14, 15]. Other novel aspects, such as the complex role of oxidative stress in the development of this malignancy, also start to gather much attention [16, 17]. Antioxidative responses are usually mounted under normal circumstances to scavenge reactive oxygen species [18]. However, this can also be manipulated by malignant cells to escape from the clearance [19]. Antioxidative stress proteins are therefore speculated to be potential therapeutic targets, too [19]. Despite the drastic development of agents targeting these molecularly altered groups, the number of patients benefiting from these regimens is nowhere near satisfying, while the resistance rate is also rising extensively [20].

The Cancer Genome Atlas program (TCGA) serves as a great resource to explore computationally novel biomarkers to characterize and stratify tumors further into subclusters with distinctive phenotypes. We noticed the altered immune infiltration landscapes in both LUAD and LUSC samples and identified clusters of tumors that showed differences in terms of immune-related gene expression and functional pathways. Unlike most of the studies that started with genotypical differences, we employed GSVA to look at curated gene set differences and reconstructed the genes afterward. The predicted response to drugs of interest for identified clusters may also shed light on future research on targeted therapy and clinical considerations of individualized treatment.

## 2. Materials and Methods

### 2.1. Data Source

RNA-sequencing (RNA-seq) matrices of LC were downloaded from the Genomic Data Commons database (GDC, https://portal.gdc.cancer.gov/). The lung adenocarcinoma and LUSC datasets were named TCGA-LUAD and TCGA-LUSC, respectively. RNA-seq count files were normalized and converted to TPM.

### 2.2. Algorithms for Immune/Stromal Infiltration Overview

Two well-developed and widely applied algorithms were employed in this study: ESTIMATE [21] and xCell [22].

### 2.3. Gene Set Variation Analyses, GSVA

One major collection from the Molecular Signature Database (MSigDB) C7: all immunologic signature gene sets were used to calculate the GSVA score for all samples in TCGA-LUAD and TCGA-LUSC, tumor, and nontumor [23]. It represents cell states and perturbations within the immune system. Its subset C7: ImmuneSigDB was also simultaneously employed. This represents chemical and genetic perturbations of the immune system generated by manual curation of published studies in human and mouse immunology.

### 2.4. Differential Analyses

Scores of each gene set generated from GSVA were compared between tumor and nontumor samples using limma package in R (FDR < 0.01, *p* < 0.01, |fold change| > 1.5) [24]. Common differentially enriched gene sets returned from both curated MSigDB collections were extracted through a Venn plot. All genes included in these gene sets were combined, and duplicates were excluded.

### 2.5. Consensus Clustering

Consensus clustering analyses were conducted with ConsensusClusterPlus [25]. Agglomerative pam clustering was performed, and Pearson correlation distances were calculated. Resampling was repeated 10 times for 80% of the samples.

### 2.6. Weighted Gene Correlation Network Analyses, WGCNA

Expression matrices of the list of genes generated from the last step were extracted from TCGA-LUAD and TCGA-LUSC. Cluster information was input as a feature for the selection of significantly connected hub genes through WGCNA. The analyses were conducted in R [26, 27]. The soft threshold *β* was determined through network topology analysis. The adjacency matrix was subsequently transformed into one topological overlap matrix (TOM), followed by the calculation of corresponding dissimilarity (1-TOM). Then, average linkage hierarchical clustering was performed based on the TOM-based dissimilarity measure. The minimum module size was set as 30. Next, the eigengene value of each module was calculated, and a cutline of 0.25 was set to merge modules for the dendrogram. The absolute value of Pearson's correlation was used to represent the connectivity of genes. Hub genes were defined as genes with high within-module connectivity (module membership over 0.8, gene significance over 0.1, and weight over 0.1).

### 2.7. Predicted Protein Interaction Network Analysis

Hub genes were entered into the Search Tool for the Retrieval of Interacting Genes/Proteins (STRING 11.5, https://string-db.org/), edges were drawn based on the strength of data support, and the confidence score was set as medium (0.4).

### 2.8. Single-Gene Gene Set Enrichment Analyses, GSEA

Tumor samples were stratified into two groups based on the high (≥50%) or low (<50%) expression of key hub genes. GSEA (version 3.0, http://software.broadinstitute.org/gsea/index.jsp) was employed to evaluate the differences between the two biological states with differently expressed key genes [28]. Another collection of C2: curated gene sets were also acquired from MSigDB (refer to GSVA method part). Functional gene sets with *p* less than 0.05 after 1000 times of sampling were considered statistically significant.

### 2.9. Chemotherapeutic Response Prediction

Expression matrices of chosen drugs were acquired from Cancer Genome Project 2016 (cgp2016). Drug response/sensitivity was reflected with the half-maximal inhibitory concentration (IC50). This was estimated by ridge regression through pRRophetic package in R [29].

## 3. Statistical Processing

Independent-sample *t*-test (comparisons of the predicted drug responses between two clusters of LUAD, for example), one-way ANOVA (comparisons of infiltration scores, overall and grouped by clinical characteristics, and comparisons of gene expression among different clusters), and chi-square or Fisher's exact test (comparisons between low versus high *LSM* level with different clinical characteristic) were performed, Bonferroni correction was applied for post hoc comparisons, two-tailed p was provided, and a value <0.05 was generally deemed statistically significant unless specified otherwise.

## 4. Results

### 4.1. The Shifted Landscape of Immune Infiltration in LUAD and LUSC in Comparison to Normal Tissue

The study design is illustrated in a flowchart (Figure 1). The clinical features of the two datasets are presented in Table 1. In the first step, with the help of two algorithms, ESTIMATE and xCell, we were able to broadly look at the purity of tumor samples and whether they possessed modified immune infiltration. The means of the three major scores reported are displayed in Figure 2 as radar plots. It was observed that calculations from both algorithms showed clearly reduced scores (*p* = 0.0019 for the stromal score reported for LUAD in xCell, *p* < 0.0001 for the rest of the comparisons) for both histological subtypes. This, in addition to the reduced relative frequencies of high scores, indicated abnormally modulated immune cell/stromal cell infiltration in LUAD and LUSC.

This drastic difference in immune/stromal infiltration intrigued us to subsequently investigate whether groups stratified by clinical characteristics within each histological type exhibit further differences. Age (older than 65 or not), gender, and overall staging were used to stratify patient groups. Major scores from ESTIMATE were compared among groups, as shown in Figure 3.

In LUAD, stromal, immune, and ESTIMATE scores varied significantly among groups of different gender and age. There were no significant differences in stromal scores among samples at different stages, but the immune score and ESTIMATE score tended to decrease as the disease progressed into later stages (Figure 3(a)).

On the other hand, LUSC showed a different pattern. In LUSC, only gender was observed to be significantly associated with infiltration scores, whereas neither age nor staging seemed to demonstrate a discrepancy in these scores (Figure 3(b)).

### 4.2. LUAD and LUSC Subgrouping Based on Immune-Related Gene Features

LUSC simply grouped by clinical characteristics did not seem to be highly heterogeneous in terms of immune/stromal infiltration, as Figure 3 showed. However, considering the existing evidence showing immune-related implications in LUSC, we explored further its potential underlying heterogeneity in immunologic features with clustering analyses, using the expression matrices from LUAD and LUSC in combination with the updated list of all immune-related genes provided by ImmPort (till December 1, 2021, https://www.immport.org). Consensus clustering revealed two distinct clusters in LUAD and three in LUSC (Figure 4). These clusters can be considered as groups with distinct immunologic patterns. The following of this study will focus on the questions of how they differ exactly and which genes or pathways contribute to these differences.

### 4.3. Mining Immune-Related Gene List That Is Differentially Regulated between Tumor and Normal Samples

WGCNA analyses were employed to identify key genes associated with the clusters acquired from previous consensus clustering. Instead of using the expression matrix of genes, we used matrices of enrichment scores of gene sets/pathways acquired by gene set variation analyses (GSVA). The analyses were performed on the original gene expression matrices of LUAD and LUSC, and enrichment scores were calculated for each sample. To further reduce the noise and increase the specificity, two series of immune-related curated gene sets (C7: all immunologic signature gene sets and C7: ImmuneSigDB gene sets) were used separately, and subsequent limma analyses were applied to find differentially enriched gene sets (DEGSs) between tumor and normal samples. For LUAD, no significantly downregulated pathways were returned based on the threshold we set while using curated gene sets from ImmuneSigDB to conduct the differential analysis; remaining overlapping DEGSs were shown in a Venn plot (Figure 5): enrichment scores of 13 gene sets were increased in LUAD which was shared between both analyses; enrichment scores of 60 gene sets were universally increased, and 5 gene sets decreased in LUSC compared to normal. The complete list of DEGSs in LUAD and LUSC is detailed in Table 1. All genes included in these differentially enriched gene sets were abstracted and combined as one list of genes for LUAD and LUSC, respectively.

The expression matrices of all genes involved in the gene sets listed in Table 2 were extracted from LUAD as well as LUSC gene expression matrices. With the cluster information identified from the previous step, the WGCNA analyses were conducted. Modules highly correlated with the clusters were identified. Hub genes which showed the highest connectivity in each relevant module were extracted additionally (Figure 6). Consequently, only one hub gene was revealed with a module membership (MM) to the blue module of 0.8085, *p* < 0.0001. On the contrary, 21 hub genes were highly connected to the brown module in LUSC, and 3 out of them (*CD74*, *GIMAP7*, and *SELPLG*) have absolute gene significance (GS) over 0.1 regarding all three clusters.

### 4.4. Differential Hub Gene Expression in LUAD and LUSC Clusters Based on WGCNA

At the protein level, currently available evidence from the STRING database indicated that the hub gene of the blue module in LUAD was isolated from the interconnected group of 21 genes in LUSC. The latter genes formed a network with significant interactions (average node degree 9.52, average local clustering coefficient 0.747, enrichment *p* < 1 × 10^−16^, Figure 7(a)).

The expression levels of *LSM2* significantly differ among two clusters of LUAD and the normal control (Figure 7(b)). A higher level of expression was observed in older patients (over 65, OR = 1.003, *p* = 0.0127). In terms of clinical features, however, it failed to be statistically involved with advanced pathological stages in LUAD (Table 3, Table 4).

The expression profile of 21 hub genes exhibited some interesting patterns (Figure 7(c)). A universal pattern of expression level as C2 < C3 < C1 < normal could be appreciated across all these genes. Levels of almost all genes in normal samples were significantly higher than any of the clusters of tumor cases, while levels of almost all genes in cluster 2 were significantly lower than any other group (Figure 7(c), Supplementary Table 1).

### 4.5. Linkage to the Clinical Picture

We predicted the sensitivity of different clusters to clinically applied therapeutical agents whose expression matrices are also available in cgp2016. We also conducted single-gene GSEA analyses to further look at possibly different functions in samples with high/low expression levels of *CD74*, *GIMAP7*, and *SELPLG*. Again, out of 21 hub genes highly connected to the brown module in LUSC, these three (*CD74*, *GIMAP7*, and *SELPLG*) had absolute gene significance and thus were chosen for this part of the analysis. It was not surprising to see a generally worse response of cluster 1 of LUAD to most agents (Figure 8(a)) since it had a higher expression of *LSM2*. One exception is the response to erlotinib: cluster 1 had a better-predicted response (Figure 8(a)). We conducted correlation analyses and observed an interesting positive correlation between the expression of *LSM2* and the response to erlotinib, in contrast to the most variable paclitaxel (Figure 9(a)). Rather intriguingly, on the note of LUSC, cluster 2, with the lowest expression profile of key hub genes, had the best-predicted responses to all agents except erlotinib (Figure 8(b)).

After conducting GSEA, we found dissimilarities between the two clusters with different expression levels of *LSM2* when it came to various functional pathways involving DNA replication and repair. On the other hand, 3 hub genes of LUSC stratified tumor samples into groups with differently altered cytokine-cytokine interaction, chemokine signaling, and cell adhesion molecules (Figure 9(b)).

## 5. Discussion

Clinical management of LC has evolved remarkably. A variety of targeted therapies in combination of chemotherapeutic regimens have emerged thanks to a better understanding of the nature of the tumor. Prolonged survival has been observed, yet the proportion of patients benefiting from available standard treatment remains low, and persistent responses could not be ensured. Patients with no currently identifiable targets, who comprise the majority, rely on chemotherapy plus certain immunotherapeutic agents such as immune checkpoint inhibitors. It remains a great challenge to find more satisfactory alternatives, if available, to maximize clinical benefit and reduce side effects as well as a financial burden.

The mainstay of this study is the identification of key hub genes acquired and refined through a series of bioinformatic pipelines. The significantly different expression profile of these genes seems to have contributed to the different responses of tumor subgroups to immunochemotherapeutic agents.

The only hub gene identified in LUAD, *LSM2*, was strongly associated with the clustering. The GSEA, based on the expression of *LSM2*, depicted the dysregulated pathways, including DNA replication, nucleotide excision repair, and mismatch repair. As a gene encoding member of the Like-Smith (*LSM*) family of RNA-binding proteins, *LSM2* has not been investigated extensively, but one other member in the *LSM* family, *LSM1*, was found to be highly related to “Chemoresistance pathways under the mediation of constitutive activation of PI3K pathway and *BCL-2* in SCLC” and “IGF-1 receptor/EGFR cooperation in LC,” suggesting a potential role in LC tumorigenesis [30]. Increased expression of *LSM1* has been found to accelerate tumor cell transformation and progression in breast cancer and mesothelioma [30–32]. It is speculated to do so by mediating U4/U6 snRNP formation and modulating the pre-mRNA splicing [33]. In our study, *LSM2* did not seem to be grossly related to the clinical features but was shown to be negatively associated with most of the agents included in the drug-response prediction, indicating a worse prognosis. The positive association between expression of *LSM2* and predicted response to erlotinib implied possible interactions with the EGFR signaling pathway; this observation necessitates further verification.

Erlotinib was permitted by the Food and Drug Administration (FDA) as early as 2004 and has existed as a second/third-line therapeutical choice for patients with advanced LC. Even though better responsiveness has been observed in adenocarcinoma [34], especially for those with a higher presence of EGFR mutation, for whom this drug was designed in the first place [35], its clinical usage was very restricted due to its low response rate, high cost, and the fact that its recommended dosage is close to its maximum tolerated dose [36]. What is more, erlotinib or erlotinib in combination with other chemotherapeutic agents such as carboplatin and paclitaxel did not differ much in terms of efficacy [37]. Secondary mutation of EGFR was speculated to be contributory to the resistance of erlotinib, yet the addition of other EGFR tyrosine kinase inhibitors (TKIs) did not seem to enhance the efficacy or counteract the resistance [38]. Two clusters with significant differences in *LSM2* expression had comparable responses to direct monoclonal EGFR-binding fragments, but drastic differences in their responses to EGFR-TKI. Based on this, we speculate that *LSM2* might be one good standard of the biomarkers that cooperatively mediated the effect of such EGFR-TK targeted agents. The evidence of reversibility of drug sensitivity indicated that nonmutational mechanisms of drug escape existed [39] and thus further supported our speculation. And not only limited to adenocarcinoma, but a portion of LUSC, such as cluster 3 identified from TCGA-LUSC, might also be able to benefit from the introduction of EGFR-TKIs into the treatment regimens. Contrarily, the best responses to most drugs were predicted in cluster 2 of LUSC, while expression levels of 21 hub genes were observed to be relatively lowest in cluster 2. These observations implied the possible effect of this refined immune-related functional gene set on the clinical response of LUSC patients.

The complex interplay between the predicted effect of TKIs and our clustering could be looked at from another aspect. Crizotinib is another typical receptor TKI in target therapy. Other similar or more potent drugs have also been developed after this first FDA-approved anaplastic lymphoma kinase (ALK) inhibitor [40]. The trend of response clusters exhibited to this drug was like the rest of the drugs analyzed, contrary to erlotinib.

It is worth mentioning the comparison of predicted responses should be considered merely as references when making decisions on combinative therapy or backbone strategy rather than selecting “the best choice.” For example, the best response observed in cluster 1 of LUAD to paclitaxel does not make it superior to etoposide. Instead, it underlies a possible complex regimen consisting of such agents or their comparable ones.

*CD74*, P-selectin glycoprotein ligand (*SELPLG*) gene, and GTPase of the immunity-associated protein (*GIMAP*) gene were three genes with the highest GS in our WGCNA analyses, differently expressed in three clusters of LUSC. *GIMAP* family members are the most highly expressed in immune cells, and GIMAP4 has been shown to be localized to the cytoskeletal system and plays a vital role in cellular transport processes [41, 42]. In our study, *GIMAP7* was shown to be a major differently expressed between cluster 1 and cluster 2 in LUSC (Figure 7(c)). It also led to different predicted responses to medications targeting microtubule functions and the cytoskeleton system. *CD74* and *SELPLG* are also all proven to be important in associating immune cells to migrate and/or adhere [43, 44]. The proper execution of these functions could contribute to the development of LUSC and influent its responses to anticancer recipes. Interestingly, CD74 also mediated the protective effect on the lung tissue in response to hyperoxia through macrophage migration inhibitory factor (MIF) [45]. In other malignancies, this MIF/CD74 axis also has been confirmed to be a potential therapeutic target [46]. Similarly, the reactive oxygen species-cancer axis has been found in a large range of malignancies, including LC, affected by various regulators such as noncoding RNAs like miR-34, miR-155, miR506, and miR-21 [47–51]. All this evidence, in addition to our findings here, indicated the importance of further exploring the dysregulated pathways related to oxidative stress in LC.

While clusters of LUSC generally showed better-predicted responses toward these agents with similar antimitotic properties (docetaxel, paclitaxel, vinblastine, vinorelbine, and gemcitabine), it is also very exciting to see the different extents across specific agents observed among the clusters. Cluster 2 has the best-predicted response to paclitaxel, while cluster 1 has the best-predicted response to docetaxel. This implied the prospect of a much more individualized selection of chemotherapeutic agents.

## 6. Conclusion

In a word, we provided a new stratification aspect for LCs based on their immune-related nature as well as key genes leading this clustering process and accompanied possible different responses to some clinically available drugs.

## Figures and Tables

**Figure 1:** Scheme of main analyses conducted in this study. TCGA: The Cancer Genome Atlas; LUAD: lung adenocarcinoma; LUSC: lung squamous cell carcinoma; ESTIMATE: Estimation of STromal and Immune cells in MAlignant Tumors using Expression data; WGCNA: Weighted Gene Correlation Network Analysis.

**Figure 2:** LUAD and LUSC exhibited shifted landscapes of immune infiltration in comparison to normal tissue. Radar plots in the first line show the means of stromal score, immune score, and ESTIMATE score reported by ESTIMATE, while their frequency distribution histograms are shown in the following lines separately (tumor versus normal tissue) for adenocarcinoma (a) and squamous cell carcinoma of the lungs (b); stromal score, immune score and microenvironment score reported by xCell were illustrated for adenocarcinoma (c) and squamous cell carcinoma (d). For comparisons of means, one-way ANOVAs were conducted, and two-tailed *p* values were calculated after Bonferroni corrections (values not shown in the figure).

**Figure 3:** LUAD and LUSC exhibited different levels of infiltration in subgroups of different clinical features: age, gender, and stages. (a) Levels of stromal score, immune score, and ESTIMATE score in different groups of LUAD, top left: age, top right: gender, bottom: stages; (b) Levels of stromal score, immune score, and ESTIMATE score in different groups of LUSC, top left: age, top right: gender, bottom: stages; independent-samples *t*-tests were applied for comparison between two groups when samples were stratified based on age or gender; one-way ANOVAs were conducted among groups stratified based on overall stages, and two-tailed *p* values were calculated after Bonferroni corrections, ^∗^*p* < 0.05, LUAD: lung adenocarcinoma, LUSC: lung squamous cell carcinoma.

**Figure 4:** Clustering analyses revealed two clusters in LUAD and three clusters in LUSC based on immunologic features. (a) LUAD; (b) LUSC; from left to right: heatmap of consensus matrix, cumulative distribution function (CDF) curve, and delta area plot.

**Figure 5:** Venn plot showing the altered enrichment of immune-related gene sets in LUAD and LUSC. (a): LUAD; (b): LUSC. ALL_Immunologic_LUAD_UP: gene sets defined in C7: all immunologic signature gene sets which had an increased enrichment score in LUAD tumor samples in comparison with normal samples; the same rule applies for the remaining group names shown in the figure.

**Figure 6:** WGCNA analyses revealed a blue module highly associated with LUAD clusters and a brown module for LUSC. (a) LUAD, with a soft threshold of 3; (b): LUSC, with a soft threshold of 7.

**Figure 7:** Expression of hub genes in different clusters of LUAD and LUSC. (a) Predicted protein interactions of hub genes constructed by STRING. LSM2 (yellow) was from LUAD, and the other 21 red nodes were from LUSC; (b) expression level of LSM2 in TCGA-LUAD samples; (c) expression level of 21 hub genes in TCGA-LUSC samples. One-way ANOVAs were conducted accordingly, and two-tailed *p* values were calculated after Bonferroni corrections, ^∗^*p* < 0.05, numbers followed by the asterisk indicate the significant differences between the group and other clusters.

**Figure 8:** Predicted response/sensitivity of different clusters of LUAD and LUSC to some common therapeutical agents. Student's *t*-tests or one-way ANOVAs were conducted accordingly, and two-tailed *p* values were calculated after Bonferroni corrections (refer to Supplementary Table 2 for detailed statistics), ^∗^*p* < 0.05, numbers followed by the asterisk indicate the significant comparisons between clusters.

**Figure 9:** Functional differences between groups with high and low expression of key hub genes. (a) Spearman correlation analyses of LSM2 expression and predicted responses of clusters in LUAD to erlotinib, in comparison with paclitaxel, 1: cluster 1, 2: cluster2; (b) gene set enrichment analyses after grouping tumor samples into high versus low expression of the major hub genes: LSM2 (LUAD), CD74, GIMAP7, and SELPLG (LUSC).

**Table 1:** Clinical characteristics of overall LUAD and LUSC samples involved in this study.

Characteristics	Levels	LUAD overall	LUSC overall
*n*		513	501
T stage, *n* (%)	T1	168 (32.9%)	114 (22.8%)
	T2	276 (54.1%)	293 (58.5%)
	T3	47 (9.2%)	71 (14.2%)
	T4	19 (3.7%)	23 (4.6%)
N stage, *n* (%)	N0	330 (65.9%)	319 (64.4%)
	N1	95 (19%)	131 (26.5%)
	N2	74 (14.8%)	40 (8.1%)
	N3	2 (0.4%)	5 (1%)
M stage, *n* (%)	M0	344 (93.2%)	411 (98.3%)
	M1	25 (6.8%)	7 (1.7%)
Pathologic stage, *n* (%)	Stage I	274 (54.3%)	244 (49.1%)
	Stage II	121 (24%)	162 (32.6%)
	Stage III	84 (16.6%)	84 (16.9%)
	Stage IV	26 (5.1%)	7 (1.4%)
Gender, *n* (%)	Female	276 (53.8%)	130 (25.9%)
	Male	237 (46.2%)	371 (74.1%)
Race, *n* (%)	Asian	7 (1.6%)	9 (2.3%)
	Black or African American	52 (11.7%)	30 (7.7%)
	White	387 (86.8%)	349 (89.9%)
Smoker, *n* (%)	No	74 (14.8%)	18 (3.7%)
	Yes	425 (85.2%)	471 (96.3%)
Age, median (IQR)		66 (59, 72.75)	68 (62, 73)
Number_pack_years_smoked, median (IQR)		40 (20.5, 50)	50 (30, 64.25)

Note: samples with missing clinical information were excluded thus contributing to different sum under different characteristic categories. IQR: interquartile range.

**Table 2:** Complete list of altered enrichment of immune-related gene sets.

LUAD
*GSE24634_TREG_VS_TCONV_POST_DAY5_IL4_CONVERSION_UP*
*GSE18893_TCONV_VS_TREG_24H_TNF_STIM_UP*
*GSE24634_TEFF_VS_TCONV_DAY5_IN_CULTURE_UP*
*GSE21063_WT_VS_NFATC1_KO_8H_ANTI_IGM_STIM_BCELL_UP*
*GSE15750_DAY6_VS_DAY10_TRAF6KO_EFF_CD8_TCELL_UP*
*GSE15750_DAY6_VS_DAY10_EFF_CD8_TCELL_UP*
*GSE39556_CD8A_DC_VS_NK_CELL_MOUSE_3H_POST_POLYIC_INJ_UP*
*GSE29614_CTRL_VS_DAY7_TIV_FLU_VACCINE_PBMC_DN*
**GSE36476_CTRL_VS_TSST_ACT_40H_MEMORY_CD4_TCELL_YOUNG_DN**
**GSE36476_CTRL_VS_TSST_ACT_72H_MEMORY_CD4_TCELL_OLD_DN**
**GSE36476_CTRL_VS_TSST_ACT_40H_MEMORY_CD4_TCELL_OLD_DN**
**GSE36476_CTRL_VS_TSST_ACT_72H_MEMORY_CD4_TCELL_YOUNG_DN**
**GSE13547_2H_VS_12_H_ANTI_IGM_STIM_BCELL_DN**

LUSC
*GSE24634_TEFF_VS_TCONV_DAY3_IN_CULTURE_UP*
*GSE19888_ADENOSINE_A3R_ACT_VS_A3R_ACT_WITH_A3R_INH_PRETREATMENT_IN_MAST_CELL_UP*
*GSE24634_TREG_VS_TCONV_POST_DAY7_IL4_CONVERSION_UP*
*GSE18893_TCONV_VS_TREG_24H_TNF_STIM_UP*
*GSE5679_CTRL_VS_RARA_AGONIST_AM580_TREATED_DC_UP*
*GSE14415_INDUCED_TREG_VS_TCONV_UP*
*GSE24634_TREG_VS_TCONV_POST_DAY3_IL4_CONVERSION_UP*
*GSE24634_TEFF_VS_TCONV_DAY5_IN_CULTURE_UP*
*GSE5679_CTRL_VS_PPARG_LIGAND_ROSIGLITAZONE_TREATED_DC_UP*
*GSE27241_WT_VS_RORGT_KO_TH17_POLARIZED_CD4_TCELL_UP*
*GSE13547_CTRL_VS_ANTI_IGM_STIM_BCELL_12H_UP*
*GSE15750_DAY6_VS_DAY10_EFF_CD8_TCELL_UP*
*GSE30962_PRIMARY_VS_SECONDARY_ACUTE_LCMV_INF_CD8_TCELL_UP*
*GSE24634_TREG_VS_TCONV_POST_DAY5_IL4_CONVERSION_UP*
*GSE39556_CD8A_DC_VS_NK_CELL_MOUSE_3H_POST_POLYIC_INJ_UP*
*GSE19888_CTRL_VS_A3R_INHIBITOR_TREATED_MAST_CELL_UP*
*GSE14415_INDUCED_TREG_VS_FAILED_INDUCED_TREG_UP*
*GSE22432_PDC_VS_TGFB1_TREATEDCOMMON_DC_PROGENITOR_UP*
*GSE15271_CXCR4_POS_VS_NEG_GC_BCELL_UP*
*GSE7764_IL15_TREATED_VS_CTRL_NK_CELL_24H_UP*
*GSE22432_MULTIPOTENT_VS_COMMON_DC_PROGENITOR_UNTREATED_UP*
*GSE13547_WT_VS_ZFX_KO_BCELL_ANTI_IGM_STIM_2H_UP*
*GSE24634_TEFF_VS_TCONV_DAY7_IN_CULTURE_UP*
*GSE21063_WT_VS_NFATC1_KO_8H_ANTI_IGM_STIM_BCELL_UP*
*GSE21360_SECONDARY_VS_TERTIARY_MEMORY_CD8_TCELL_UP*
*GSE15750_DAY6_VS_DAY10_TRAF6KO_EFF_CD8_TCELL_UP*
*GSE7568_IL4_VS_IL4_AND_DEXAMETHASONE_TREATED_MACROPHAGE_UP*
***GSE29618_MONOCYTE_VS_MDC_DAY7_FLU_VACCINE_UP***
***GSE11057_PBMC_VS_MEM_CD4_TCELL_UP***
**GSE36476_CTRL_VS_TSST_ACT_40H_MEMORY_CD4_TCELL_YOUNG_DN**
**GSE17974_0H_VS_24H_IN_VITRO_ACT_CD4_TCELL_DN**
**GSE16450_IMMATURE_VS_MATURE_NEURON_CELL_LINE_DN**
**GSE36476_CTRL_VS_TSST_ACT_72H_MEMORY_CD4_TCELL_YOUNG_DN**
**GSE14415_TCONV_VS_FOXP3_KO_INDUCED_TREG_DN**
**GSE25088_WT_VS_STAT6_KO_MACROPHAGE_IL4_STIM_DN**
**GSE36476_CTRL_VS_TSST_ACT_40H_MEMORY_CD4_TCELL_OLD_DN**
**GSE36476_CTRL_VS_TSST_ACT_72H_MEMORY_CD4_TCELL_OLD_DN**
**GSE33292_WT_VS_TCF1_KO_DN3_THYMOCYTE_DN**
**GSE24574_BCL6_LOW_TFH_VS_TCONV_CD4_TCELL_DN**
**GSE21927_SPLEEN_C57BL6_VS_EL4_TUMOR_BALBC_MONOCYTES_DN**
**GSE14415_NATURAL_TREG_VS_TCONV_DN**
**GSE15930_NAIVE_VS_48H_IN_VITRO_STIM_CD8_TCELL_DN**
**GSE22886_NAIVE_CD4_TCELL_VS_48H_ACT_TH1_DN**
**GSE411_100MIN_VS_400MIN_IL6_STIM_MACROPHAGE_DN**
**GSE10239_NAIVE_VS_DAY4.5_EFF_CD8_TCELL_DN**
**GSE22886_UNSTIM_VS_STIM_MEMORY_TCELL_DN**
**GSE22886_UNSTIM_VS_IL2_STIM_NKCELL_DN**
**GSE17974_CTRL_VS_ACT_IL4_AND_ANTI_IL12_24H_CD4_TCELL_DN**
**GSE13547_2H_VS_12_H_ANTI_IGM_STIM_BCELL_DN**
**GSE14415_INDUCED_VS_NATURAL_TREG_DN**
**GSE21546_ELK1_KO_VS_SAP1A_KO_AND_ELK1_KO_DP_THYMOCYTES_DN**
**GSE3982_MEMORY_CD4_TCELL_VS_TH2_DN**
**GSE24634_NAIVE_CD4_TCELL_VS_DAY5_IL4_CONV_TREG_DN**
**GSE21546_UNSTIM_VS_ANTI_CD3_STIM_DP_THYMOCYTES_DN**
**GSE22886_UNSTIM_VS_IL15_STIM_NKCELL_DN**
**GSE21546_WT_VS_ELK1_KO_ANTI_CD3_STIM_DP_THYMOCYTES_DN**
**GSE15930_NAIVE_VS_48H_IN_VITRO_STIM_IFNAB_CD8_TCELL_DN**
**GSE15930_NAIVE_VS_48H_IN_VITRO_STIM_IL12_CD8_TCELL_DN**
**GSE22886_NAIVE_CD4_TCELL_VS_12H_ACT_TH1_DN**
**GSE15930_NAIVE_VS_24H_IN_VITRO_STIM_CD8_TCELL_DN**
**GSE15930_NAIVE_VS_24H_IN_VITRO_STIM_INFAB_CD8_TCELL_DN**
***GSE10325_BCELL_VS_MYELOID_DN***
***GSE22886_NAIVE_TCELL_VS_MONOCYTE_DN***
***GSE10325_LUPUS_BCELL_VS_LUPUS_MYELOID_DN***

Note: the original up/down trends were in italic/bold fonts, respectively; the up/down trends revealed consistently by GSVA (as Figure 5 shows) were underlined/in bold-italic emphasis, respectively.

**Table 3:** Clinical features of LUAD patients classified by *LSM2* levels.

Feature	Levels	Low *LSM2* level	High *LSM2* level	*p*
*n*		256	257	
T stage, *n* (%)	T1	94 (18.4%)	74 (14.5%)	0.167
	T2	129 (25.3%)	147 (28.8%)	
	T3	25 (4.9%)	22 (4.3%)	
	T4	7 (1.4%)	12 (2.4%)	
N stage, *n* (%)	N0	172 (34.3%)	158 (31.5%)	0.448
	N1	41 (8.2%)	54 (10.8%)	
	N2	36 (7.2%)	38 (7.6%)	
	N3	1 (0.2%)	1 (0.2%)	
M stage, *n* (%)	M0	157 (42.5%)	187 (50.7%)	0.132
	M1	7 (1.9%)	18 (4.9%)	
Pathologic stage, *n* (%)	Stage I	146 (28.9%)	128 (25.3%)	0.140
	Stage II	57 (11.3%)	64 (12.7%)	
	Stage III	41 (8.1%)	43 (8.5%)	
	Stage IV	8 (1.6%)	18 (3.6%)	
Gender, *n* (%)	Female	145 (28.3%)	131 (25.5%)	0.231
	Male	111 (21.6%)	126 (24.6%)	
Race, *n* (%)	Asian	3 (0.7%)	4 (0.9%)	0.659
	Black or African American	30 (6.7%)	22 (4.9%)	
	White	199 (44.6%)	188 (42.2%)	
Smoker, *n* (%)	No	43 (8.6%)	31 (6.2%)	0.184
	Yes	208 (41.7%)	217 (43.5%)	
Age, median (IQR)		67 (59, 74)	65 (59, 71)	0.234
Number_pack_years_smoked, median (IQR)		36 (20, 50)	40 (25, 52)	0.337

^#^Chi-square tests were applied for T stage, M stage, pathological stage, gender, and age (>65 or ≤65); Fisher's exact test was applied for N stage; Wilcoxon signed rank test for age (median); IQR: interquartile range.

**Table 4:** Single-gene logistic regression analyses for LSM2.

Features	Total (*N*)	Odds ratio (OR)	*p*
Pathologic stage (stage III and stage IV vs. stage I and stage II)	505	0.9991 (0.995-1.002)	0.5912
Gender (male vs. female)	513	1.001 (0.998-1.003)	0.5512
Age (>65 vs. ≤65)	513	1.003 (1.001-1.006)	0.0127

## Data Availability

The labeled dataset used to support the findings of this study are available from the corresponding author upon request.

## Supplementary Materials

Supplementary 1 Supplementary Table 1: statistics of Figure 7(c). Levels of almost all genes in normal samples were significantly higher than any of the clusters of tumor cases, while levels of almost all genes in cluster 2 were significantly lower than any other group (Figure 7(c), Supplementary Table 1).

Supplementary 2 Supplementary Table 2: statistics of Figure 8. Student's *t*-tests or one-way ANOVAs were conducted accordingly, and two-tailed *p* values were calculated after Bonferroni corrections (refer to Figure 8).
